# Artificial Intelligence-Based MRI in Diagnosis of Injury of Cranial Nerves of Premature Infant and Its Correlation with Inflammation of Placenta

This article has been retracted.

**DOI:** 10.1155/2022/4550079

**Published:** 2022-03-27

**Authors:** Gui Liao

**Affiliations:** Department of Pediatrics, The Third People's Hospital of Yunnan Province, Kunming 650011, Yunnan, China

## Abstract

The study focused on the effects of artificial intelligence algorithms in magnetic resonance imaging (MRI) for diagnosing cranial nerve inflammation of placenta and the correlation between cranial nerve injury with placental inflammation was explored. The subjects were selected from 132 premature infants in the hospital. According to the pathological examination of placenta, 81 cases with chorioamnionitis were taken as the experimental group and 51 cases without chorioamnionitis were taken as the control group. The incidence of cranial nerve injury in different groups of premature infants was analyzed by MRI diagnosis based on the principal component analysis (PCA) artificial intelligence algorithm, so as to analyze the correlation between cranial nerve injury and placental inflammation in premature infants. It was found that when the PCA artificial intelligence algorithm was incorporated into MRI examination of cranial nerve injury of premature infant, the *A* (accuracy), *P* (precision), *R* (recall), and *F*1 values under the PCA algorithm were 92%, 93.75%, 90%, and 92.87%, respectively. The *A*, *P*, *R*, and *F*1 of the control group were 54%, 54.1%, 52%, and 53.03%, respectively; there were statistically significant differences between the two groups, *P* < 0.05. As for the correlation of placental inflammation and cranial nerve injury, the positive detection rate of the experimental group was 53.09%, and the positive detection rate of the control group was 15.69%, and the difference was statistically significant, *P* < 0.05. In conclusion, the PCA artificial intelligence algorithm has high effectiveness and high accuracy in auxiliary diagnosis of premature brain nerve injury, and placental inflammation greatly increases the chance of premature infant suffering from brain nerve injury.

## 1. Introduction

Premature infant refers to live-born babies with a gestational age less than 37 weeks, weighed less than 2.5 kg [1], and having a head circumference of 33 cm or less. Its organ function and adaptability are relatively poor compared to full-term premature infant, and some organs are immature [2]. It has been found that except for perinatal hypoxia-ischemia or asphyxia, hyperbilirubinemia, and hypoglycemia, cranial nerve injury is also related to premature infant placental inflammation [3, 4]. There are many types of placental inflammation, and chorioamnionitis is a common one [5, 6]. It results from pathogens infecting the chorion, amniotic membrane, and decidua of the placenta. Morphologically, it manifests as neutrophils infiltrating the villi membrane [7, 8]. Maternal chorioamnionitis can cause fetal inflammatory response syndrome, which is a subclinical state caused by the activation of the fetal immune system and release of a large number of inflammatory factors (IL-6, IL-1, IL-8, and TNF-*α*). These inflammatory factors can interfere with the normal expression of fetal brain cytokines, leading to brain damage in premature infants [9].

In recent years, although the survival rate of premature infant has increased, the probability of cranial injury has also increased. Currently, cranial injury of premature infant is mainly diagnosed by doctors assisted by imaging examination. The commonly used imaging examination methods include ultrasound, electronic computed tomography (CT), and magnetic resonance imaging (MRI). CT image has limited resolution [10], and the radiation will do harm to people's health. Hence, it is not recommended. Ultrasound examination is safe and has high repeatability, and it can dynamically observe the progress of the disease, but it has many shortcomings [11]. MRI is an advanced medical imaging examination method introduced in the early 1980s, which combines the latest research results in the fields of biology [12, 13], chemistry, physics, and medicine [14, 15]. Additionally, it is sensitive to motion and prone to artifacts [16, 17].

MRI can accurately, sensitively and noninvasively reflect the location, scope, and histological basis of brain lesions, and it is a well-recognized imaging examination method to evaluate cranial injury of premature infant. Incorporating intelligent algorithms into MRI imaging can effectively improve its shortcomings and better assist doctors in diagnosing cranial injury of premature infant. Principal component analysis (PCA) is a common data analysis method. It is often used for dimensionality reduction of high-dimensional data and can improve the quality of MRI images by extracting the main feature components of the data, thus elevating the accuracy of diagnosis [18, 19]. Leviton et al. [20] introduced the main analysis algorithm of multivariate statistical analysis into brain nerve injury and adopted statistical pattern recognition brain image feature extraction, which greatly simplified the calculation.

There have been a large number of reports of cranial injury of premature infant, but there are not many studies on placental inflammation [21, 22]. To prevent and diagnose cranial injury of premature infant caused by placental inflammation, the correlation between cranial nerve injury and placental inflammation was analyzed through MRI based on PCA, expected to provide reference for the clinical prevention, diagnosis, and treatment of cranial nerve injury of premature infant.

## 2. Materials and Methods

### 2.1. Research Subjects and Grouping

The subjects were selected from 132 premature infants in the hospital from April 2018 to April 2020. According to the pathological examination of placenta, 81 cases with chorioamnionitis were taken as the experimental group and 51 cases without chorioamnionitis were taken as the control group. The incidence of cranial nerve injury in different groups of premature infants was analyzed by MRI diagnosis based on the principal component analysis (PCA) artificial intelligence algorithm, so as to analyze the correlation between cranial nerve injury and placental inflammation in premature infants. Placental inflammation was divided into stage 0, stage I, stage II, and stage III. The study had been approved by the ethics committee of hospital, and the subjects and their family members understood the content of the study and signed an informed consent form.

Inclusion criteria were as follows: premature infants with a gestational age less than 37 weeks, the bodyweight was under 2.5 kg, and the head circumference was under 33 cm.

Exclusion criteria were as follows: premature infant with congenital malformations, those with chromosomal abnormalities and metabolic genetic diseases, and those with craniocerebral abnormalities confirmed by prenatal examination.

### 2.2. Pathological Examination of Placental Inflammation

After delivery of premature infants, 3 × 3 cm fetal membrane tissue was taken from the placenta tear as the center to make fetal membrane rolls, and then, samples were taken from the center, middle, and edge of the placenta. Amniotic membrane, chorionic plate, villi, and decidua were selected. Specimens were fixed with 10% formaldehyde, embedded in paraffin, sliced, stained with hematoxylin-eosin (H&E), and read by experienced physicians in the department of pathology.

### 2.3. Staging Diagnostic Criteria of Placental Inflammation

Placental histology is mainly chorioamnionitis (HCA), that is, maternal neutrophils infiltrate into amniotic membrane, chorion, and decidua. Inflammation stages are as follows. Stage 1: neutrophil infiltration is less and scattered, almost all confined to the chorionic space. Stage 2: neutrophil infiltration increased and extended to the chorionic plate in the chorionic tissue, but did not enter the amniotic membrane. Stage 3: neutrophils infiltrated into amniotic epithelial cells. Stages represent the progress of the disease.

### 2.4. Principal Component Analysis Artificial Intelligence Algorithm

The mathematical derivation of PCA can be carried out from the two aspects of maximum separability and nearest reconstruction. The optimization condition of the former is that the variance is the largest after division, and the optimization condition of the latter is that the distance from the point to the division plane is the smallest. This study is from the perspective of maximum separability. The inner product of two vectors *A* and *B* is expressed as follows.

(1) $$\begin{array}{c} \left(a_{1},a_{2},\ldots ,a_{n}\right)\cdot {\left(b_{1},b_{2},\ldots ,ab_{n}\right)}^{T}=a_{1}b_{1},a_{2}b_{2},\ldots ,a_{n}b_{n}. \end{array}$$

The inner product operation maps two vectors to real numbers. Geometrically, assuming that *A* and *B* are two-dimensional vectors expressed as follows, its geometric representation is shown in Figure 1.

(2) $$\begin{array}{c} A=\left(X_{1},Y_{1}\right);B=\left(X_{2},Y_{2}\right)\\ A\cdot B=\left|A\right|\left|B\right|\text{cos}b. \end{array}$$

The inner product of *B* and *A* is equal to the projection length from *B* to *A* multiplied by the modulus of *B*. Assuming that the modulus of *A* is 1, namely, ∣*A*∣ = 1, as shown in equation (4), the inner product of *B* and *A* is equal to the scalar size of *B* projected to the line where *A* is located.

(3) $$\begin{array}{c} A\cdot B=\left|B\right|\text{cos}b. \end{array}$$

In the coordinate system, the vector (3, 2) defined as the projection on the *x*-axis is 3 and the projection on the *y*-axis is 2. The projection is scalar, which can be negative. Therefore, for the vector (3, 2), to find its coordinates under (1, 0) (0, 1), it is just needed to solve the inner product. Above, to describe a vector accurately, a set of bases is determined first and then the projection value on each line where the basis is located is given. For the sake of convenience, the modulus length of the group basis vector is generally taken as 1, so that the inner product can directly represent the projection. For the vector (3, 2), the new coordinates in the group base is calculated as given in the following equation, which can be expressed by matrix multiplication.

(4) $$\begin{array}{c} \left(\begin{array}{cc} \frac{1}{\sqrt{2}} & \frac{1}{\sqrt{2}}\\ -\frac{1}{\sqrt{2}} & \frac{1}{\sqrt{2}} \end{array}\right)\left(\begin{array}{c} 3\\ 2 \end{array}\right)=\left(\begin{array}{c} 5\sqrt{2}\\ -\frac{1}{\sqrt{2}} \end{array}\right). \end{array}$$

The two rows of the left matrix are two bases, which are multiplied by the original vector to obtain the new base coordinates. If there are *m* two-dimensional vectors, they are arranged into a two-row *m*-column matrix, which is multiplied by the base matrix to get the value under the new base. For data points (1, 1), (2, 2), and (3, 3), the equation is expressed as follows.

(5) $$\begin{array}{c} \left(\begin{array}{cc} \frac{1}{\sqrt{2}} & \frac{1}{\sqrt{2}}\\ -\frac{1}{\sqrt{2}} & \frac{1}{\sqrt{2}} \end{array}\right)\left(\begin{array}{ccc} 1 & 2 & 3\\ 1 & 2 & 3 \end{array}\right)=\left(\begin{array}{ccc} \frac{2}{\sqrt{2}} & \frac{4}{\sqrt{2}} & \frac{6}{\sqrt{2}}\\ 0 & 0 & 0 \end{array}\right). \end{array}$$

The general representation is as the following equation, where *P*_*i*_ is a row vector, which represents the *i*^th^ basis, and *A*_*j*_ is a column vector, which represents the *j*^th^ original data.

(6) $$\begin{array}{c} \left(\begin{array}{c} P_{1}\\ \begin{array}{c} P_{2}\\ \vdots \\ P_{R} \end{array} \end{array}\right)\left(a_{1},a_{2},\ldots ,a_{m}\right)=\left(\begin{array}{cccc} P_{1}a_{1} & P_{1}a_{2} & \ldots & P_{1}a_{m}\\ P_{2}a_{1} & P_{2}a_{2} & \ldots & P_{2}a_{m}\\ \vdots & \vdots & \vdots & \vdots \\ P_{R}a_{1} & P_{R}a_{1} & \ldots & P_{R}a_{m} \end{array}\right). \end{array}$$

To multiply two matrices is to transform each column vector in the right matrix into each row vector in the left matrix. In other words, a matrix can represent a linear transformation. Variance describes the degree of dispersion of the value, and the variance of the variable is expressed as follows.

(7) $$\begin{array}{c} \text{Var}\left(a\right)=\frac{1}{m}{\sum_{i=1}^{m}\left(a_{i}-\mu \right)}^{2}. \end{array}$$

If the variable mean is 0, the variance can be expressed by the sum of squares of the elements divided by the number of elements, as shown in the following equation.

(8) $$\begin{array}{c} \text{Var}\left(a\right)=\frac{1}{m}\sum_{i=1}^{m}a_{i}{}^{2}. \end{array}$$

One-dimensional space uses variance to indicate the degree of data dispersion. In order to allow the two variables to represent the original information as much as possible, it is a must that there is no linear correlation between them. The covariance is expressed as follows.

(9) $$\begin{array}{c} Cov\left(a,b\right)=\frac{1}{m-1}\sum_{i=1}^{m}\left(a_{i}-\mu_{a}\right)\left(b_{i}-\mu_{b}\right). \end{array}$$

Since the mean value is 0, the covariance is calculated as given in equation (10). A covariance of 0 means that the two variables are linearly uncorrelated. For the covariance to be 0, the second basis is selected in the direction orthogonal to the first basis. The dimensionality reduction optimization is to reduce *n*-dimensional vectors to *K*-dimensional.

The ultimate result is related to the variance within the variables and the covariance between variables. Both can be expressed in the form of inner product, and the inner product is related to the matrix multiplication. Assuming there are only two variables, *a* and *b*, they form a matrix by rows, as shown in equation (11).

(10) $$\begin{array}{c} Cov\left(a,b\right)=\frac{1}{m}\sum_{i=1}^{m}a_{i}b_{i}, \end{array}$$

(11) $$\begin{array}{c} X=\left(\begin{array}{cccc} a_{1} & a_{2} & \ldots & a_{m}\\ b_{1} & ab_{2} & \ldots & b_{m} \end{array}\right). \end{array}$$

The diagonals of the matrix are the variances of the two variables, and the other elements are the covariances of *a* and *b*. The two are included in a matrix, as shown in the following equation.

(12) $$\begin{array}{c} \frac{1}{m}XX^{T}=\left(\begin{array}{cc} \frac{1}{m}\sum_{i=1}^{m}a_{i}{}^{2} & \frac{1}{m}\sum_{i=1}^{m}a_{i}b_{i}\\ \frac{1}{m}\sum_{i=1}^{m}a_{i}b_{i} & \frac{1}{m}\sum_{i=1}^{m}b_{i}{}^{2} \end{array}\right). \end{array}$$

To deduce, if there are *m* and *n*-dimensional data and they are arranged in a matrix *X*_*n*,*m*_, as shown in equation (13), *C* is a symmetric matrix.

(13) $$\begin{array}{c} C=\frac{1}{m}XX^{T}. \end{array}$$

According to the optimization conditions, the other elements except the diagonal are 0, and the elements are arranged on the diagonal by size from top to bottom. To describe the relationship between the original matrix and the matrix covariance matrix after the basis transformation, let the covariance matrix corresponding to the original data matrix *X* be *C*, and *P* is a set of matrixes. Let *Y* = *PX*, then *Y* is the data after base transformation of *P* by *X*. Supposing the covariance matrix of *Y* is *D*, the relationship between *D* and *C* is derived as follows.

(14) $$\begin{array}{c} D=\frac{1}{m}YY^{T}\\ =\frac{1}{m}\left(PX\right){\left(PX\right)}^{T}\\ =\frac{1}{m}PXX^{T}P^{T}\\ =P\left(\frac{1}{m}XX^{T}\right)P^{T}\\ =PCP^{T}. \end{array}$$

Then, it is necessary to complete the diagonalization. It is known that the covariance matrix *C* is a symmetric matrix. As is well-known, the eigenvectors corresponding to different eigenvalues of the real symmetric matrix must be orthogonal. Let the eigenvector *λ* multiplicity be *λ*; then, there must be *r* linearly independent eigenvectors corresponding to *λ*, so the *r* eigenvector units can be orthogonalized. Therefore, a real symmetric matrix with *n* rows and *n* columns is formed. Supposing these *n* eigenvectors are *e*_1_, *e*_2_,…, *e*_*n*_, and they are arranged by columns: *E* = (*e*_1_, *e*_2_,…, *e*_*n*_). Then, the covariance matrix *C* is expressed as follows.

(15) $$\begin{array}{c} E^{T}CE=\wedge =\left(\begin{array}{c} \begin{array}{cc} \lambda_{1} & \lambda_{1}\\ \ddots & \lambda_{1} \end{array} \end{array}\right), \end{array}$$

where ∧ is a diagonal matrix, and its diagonal elements are the eigenvalues corresponding to each eigenvector, so that *P* is obtained. *P* is the matrix arranged in rows after the eigenvectors of the covariance matrix are unitized, expressed as in equation (17). If *P* is arranged according to the eigenvalues in ∧ from large to small, then the original data matrix *X* is multiplied by the matrix composed of the first *K* rows of *P* to obtain the data matrix *Y* after dimensionality reduction.

(16) $$\begin{array}{c} P=E^{T}. \end{array}$$

Figure 2 is a flowchart of the algorithm.

### 2.5. MRI Examination

Routine preparation was carried out before MRI examination, which was generally carried out in the infants' natural sleep state. Premature infants who underwent MRI were given 2 *μ*g/kg dexmedetomidine intravenously within 10 min, and 1-2 *μ*g/(kg·h) was the maintenance dose. During examination, the cotton quilt was wrapped to keep warm, and patients with severe symptoms were provided with oxygen bag nasal mask. 3.0 T MRI and corresponding workstation, 8-channel orthogonal head coil, sequence, and imaging parameters were as follows: TlWI : FSE sequence, FOV: 18 × 18, TR/TE: 500/11 ms, matrix: 320 × 192; T2WI : FSE sequence, FOV: 18 × 18, TR/TE: 4780/100 ms, matrix: 320 × 192, excitation times 3NEX, and layer thickness/spacing: 4.0/0.5 mm. MRI images of all the infants were retrospectively analyzed by 2 radiologists who were unaware of the clinical manifestations and follow-up results using a double-blind method.

### 2.6. Evaluation Index

The PCA-processed MRI images were evaluated with the cranial nerve injury as a positive case and the healthy patient as a negative case. True positive (TP) means that the prediction is a positive case, and the actual case is also positive. False positive (FP) means that the prediction is a positive case, and the actual is a negative case. False negative (FN) means that the prediction is a negative case, and the actual is a positive case. True negative (TN) means that the prediction is a negative case, and the actual is a negative case.

(17) $$\begin{array}{c} A=\frac{\text{TN}+\text{TP}}{\text{TN}+\text{TP}+\text{FP}+\text{FN}}, \end{array}$$

(18) $$\begin{array}{c} P=\frac{\text{TP}}{\text{TP}+\text{FP}}, \end{array}$$

(19) $$\begin{array}{c} R=\frac{\text{TP}}{\text{TP}+\text{FN}}. \end{array}$$

In this study, accuracy (*A*) is used to indicate the proportion of correct predictions, calculated as given in equation (17), precision (*P*) indicates the ratio of actual positive cases among positive predictions, calculated as given in equation (18), and recall (*R*) is the ratio of the correctly predicted positive cases to all positive cases, calculated as given in equation (19).

(20) $$\begin{array}{c} F=\frac{\left(\alpha^{2}+1\right)P\times R}{\alpha^{2}\left(P+R\right)}, \end{array}$$

(21) $$\begin{array}{c} F_{1}=\frac{2P\times R}{P+R}. \end{array}$$

When the *P* index and the *R* index are contradictory, the weighted harmonic average of *P* and *R* is used, that is, the *F*-measure method, expressed as follows. When the parameter *α* = 1, it is the common *F*1, as shown in equation (21). A higher *F*1 value means the higher effectiveness of the algorithm. In an experiment to analyze the correlation between cranial injury of premature infant and placental inflammation, the positive detection rate is the ratio of the number of premature infants with cranial injury to the total number of cases multiplied by 100%.

### 2.7. Statistical Analysis

The research data were processed by SPSS version 19.0 statistical software. The collected measurement data were expressed as mean ± standard deviation ($\overset{–}{x}$ ± *s*), and the count data were expressed by percentage (%). Pairwise comparison was performed by analysis of variance, and logistic regression was used to analyze the relationship between placental inflammation stage and the risk of brain injury in premature infants. Logistic regression analysis was used to analyze the relationship between placental inflammation stage and the risk of brain injury in premature infants, and *P* < 0.05 was a threshold for significance.

## 3. Results

### 3.1. MRI Image of Premature Infant with Cranial Nerve Injury

Figures 3–5 show the MRI images of three premature infants with cranial nerve injury.  Figure 3 shows MRI images of a premature infant with mild hypoxic-ischemic encephalopathy (HIE). It was noted that the capillary endothelium was damaged and the permeability increased; and hypoxia led to the capillary reactive hyperemia and selective nerve necrosis.

Figure 4 shows MRI images of a premature infant with moderate HIE. It was noted that hypoxia led to congestion and expansion. The blood vessel development was immature, and basement membrane was damaged. Histologically, red blood cells and plasma proteins were exuded.

Figure 5 shows the MRI images of a premature infant with severe HIE. It was noted that the subcortical tissue was necrotic and brain atrophy occurred.

### 3.2. PCA Effectiveness Analysis

After MRI images of cranial nerve injury of premature infant were processed by the PCA algorithm, TP, FP, FN, and TN were 45, 3, 5, and 47, respectively; and when the control group was used for diagnosis, TP, FP, FN, and TN were 26, 22, 24, and 28, respectively, and the differences were statistically significant (*P* < 0.05).  Figure 6 shows the comparison chart of the positive and negative cases of the two.

Figure 7 shows the results of *A*, *P*, and *R*. It was noted that *A*, *P*, and *R* of PCA-based MRI were 92%, 93.75%, and 90%, respectively; and the *A*, *P*, and *R* of the control group were 54%, 54.1%, and 52%, respectively, and the differences were statistically significant (*P* < 0.05). Obviously, the three indexes of the PCA-based MRI were better versus the control group.

As shown in Figure 8, the *F*1 value of the PCA algorithm was 92.87% and the F1 value of the control group was 53.03%. Obviously, the *F*I value of the PCA algorithm was significantly higher than the control group, and there were statistically significant differences, *P* < 0.05.

### 3.3. Positive Detection Rate of Cerebral Nerve Injury in Premature Infants with Placental Inflammation

As shown in Figure 9, in the experimental group of 81 patients with chorioamnionitis, there were 43 patients with cranial nerve injury, and the positive detection rate was 53.09%, and of 51 patients without chorioamnionitis in the control group, 8 had cranial nerve injury, and the positive detection rate was 15.69%. Obviously, there were statistically significant differences in the positive detection rate of the two groups, *P* < 0.05.

### 3.4. Correlation between Cerebral Nerve Injury and Placental Inflammation Stages in Premature Infants

Figure 10 shows the pathological sections of placental inflammation in premature infants. Logistic regression analysis showed that stage II and stage III of placental inflammation were risk factors for brain nerve injury in premature infants, as given in Table 1.

## 4. Discussion

There are many factors that will cause cranial nerve injury. Clinically, MRI is generally used to assist doctors in diagnosis [23]. It has good resolution for soft tissue and high contrast. The multiparameter and multiplane imaging technology is superior in positioning and quantification. It is a noninvasive method and has no radiation damage, without the need to use contrast agents. When MRI images are processed by the PCA algorithm, the sampling density is increased and the dimensionality is reduced by discarding some information. It is an important means to alleviate the dimensional disaster [24]. When the data are affected by noise, discarding the eigenvectors corresponding to the smallest eigenvalues can reduce noise to a certain extent because they are related to noise. PCA retains the main information [25] and may discard some seemingly useless information, but these seemingly useless information happens to be important information, so PCA may aggravate overfitting. PCA also makes the features of the data after dimensionality reduction independent of each other.

In this study, the application of the PCA algorithm in MRI diagnosis of cranial nerve injury of premature infant was analyzed, and the correlation between cranial nerve placental inflammation was explored, expected to provide reference for clinical prevention, diagnosis, and treatment of cranial nerve injury of premature infant. It was found that when the PCA algorithm was incorporated in MRI examination of cranial nerve injury of premature infant, the *A*, *P*, and *R* values of the PCA algorithm were 92%, 93.75%, and 90%, respectively, and the *A*, *P*, and *R* values of the control group were 54%, 54.1%, and 52%; the diagnosis accuracy rate under the artificial intelligence algorithm was higher, which is more conducive to the diagnosis of doctors. The *F*1 value of the PCA algorithm was 92.87%, and the *F*1 value of the control group was 53.03%. Obviously, the *F*I value of the PCA algorithm was significantly higher than the control group, and there were statistically significant differences, *P* < 0.05. As for the correlation between placental inflammation and cranial nerve injury, there were 43 patients with cranial nerve injury in the experimental group, with a positive detection rate of 53.09%, and of 51 patients without chorioamnionitis in the control group, 8 had cranial nerve injury, and the positive detection rate was 15.69%. Obviously, there were statistically significant differences in the positive detection rate of the two groups, *P* < 0.05, indicating that placental inflammation would greatly increase the chance of premature infant suffering from cranial nerve injury, and it was consistent with the results of Jablonska et al. [26].

Wu et al. [27] reported that hemodynamic disturbance after intrauterine infection may be related to the release of a large number of proinflammatory cytokines. These proinflammatory cytokines can eventually lead to brain injury by influencing the formation of microglia, oligodendrocytes, astrocytes, and myelin sheath, inducing other cytokines to produce cell damage, and mediating the neurotoxicity of nitric oxide and the cytotoxicity of excitatory amino acids. Rudie et al. [28] reported that based on the diagnosis of artificial intelligence MRI, the incidence of intraventricular hemorrhage in premature infants with chorioamnionitis in pregnant mothers can reach 16.1%, and the risk of intraventricular hemorrhage can be increased by 3.2 times due to placental inflammation and the third stage of inflammation. This study found that the second and third stage inflammation of placenta was a risk factor of brain injury in premature infants, which was consistent with the literature report.

## 5. Conclusion

In this study, the PCA artificial intelligence algorithm was incorporated into MRI examination of cranial nerve injury of premature infant, and its influence on MRI images was analyzed. Then, the correlation between cranial nerve injury with placenta inflammation was explored. It was found that the PCA algorithm demonstrates a high accuracy rate, and placental inflammation will greatly increase the chance of premature infant suffering from brain nerve injury. However, shortage of this study lies in the selection of sample size that is less and not considering premature infant brain injury caused by intrauterine infection, which may affect the result of the experiment, the sample, so in a follow-up experiment, it needs to expand further comprehensive analysis based on the artificial intelligence algorithm of MRI diagnosis of premature cranial nerve injury and its correlation with placental inflammation. The sample should be expanded in subsequent experiments to strengthen the findings of the study. In conclusion, this study provides reference for clinical prevention, diagnosis, and treatment of cranial nerve injury of premature infant.

## Figures and Tables

**Figure 1:** Vector geometry representation.

**Figure 2:** The flowchart of the PCA algorithm.

**Figure 3:** MRI images of mild HIE. (a)–(c) Images of transverse, sagittal, and coronal positions, respectively.

**Figure 4:** MRI images of moderate HIE. (a)–(c) Images of transverse, sagittal, and coronal positions, respectively.

**Figure 5:** MRI images of severe HIE. (a)–(c) Images of transverse, sagittal, and coronal positions, respectively.

**Figure 6:** Comparison of positive and negative cases between PCA-based MRI and the control group.  ^*∗*^Statistically significant difference compared with the control group (*P* < 0.05).

**Figure 7:** Comparison of *A*, *P*, *R* values between PCA-based MRI and the control group.  ^*∗*^Statistically significant difference compared with the control group (*P* < 0.05).

**Figure 8:** Comparison of *F*1 values between the PCA algorithm and the control group. ^*∗*^*F*1 value of the PCA algorithm was significantly different from that of the control group (*P* < 0.05).

**Figure 9:** Comparison of positive detection rate between the experimental group and the control group.  ^*∗*^Positive detection rate of the experimental group was significantly different from that of the control group (*P* < 0.05).

**Figure 10:** Stages of inflammation in pathological sections of placental tissue (H&E staining, ×200). (a) Stage 0, normal chorionic amniotic tissue. (b) In stage I, a few neutrophils infiltrate into the subchorionic amniotic membrane. (c) In stage II, moderate neutrophils infiltrate into the subchorionic amniotic membrane. (d) In stage III, a large number of neutrophils infiltrate into the lower layer of the chorionic amniotic membrane and parts of the amniotic epithelial cells are necrotic and fall off.

**Table 1:** Analysis of placental inflammation stage and risk of cerebral nerve injury in premature infants.

Inflammation of the placenta	Cases	Incidence probability of cerebral nerve injury (%)	OR	95% CI	*P*
Stage 0	51	4.25	1	—	—
Stage I	45	34.09	2.274	0.815–6.594	0.084
Stage II	39	29.55	5.267	1.256–18.952	0.002
Stage III	7	3.03	12.345	2.314–73.264	0.002

## Data Availability

The data used to support the findings of this study are available from the corresponding author upon request.
